# Influence and Analysis of Music Teaching Environment Monitoring on Students' Mental Health Using Data Mining Technology

This article has been retracted.

**DOI:** 10.1155/2022/1120156

**Published:** 2022-10-06

**Authors:** Xinlei Dong, Xin Kang, Xiaolei Ding

**Affiliations:** ^1^School of Biology and Food Engineering, Changshu Institute of Technology, Jiangsu 215500, China; ^2^Rovira I Virgili University, Tarragona 43001, Spain; ^3^Linyi Longteng Primary School, Shandong 276000, China

## Abstract

Students currently mostly experience psychological issues like worry and fear, which are primarily brought on by the high demands placed on them. One psychotherapy technique is music therapy. The goal is to use music to enhance health, particularly as a tool to break down barriers both inside and outside the body. Based on data mining (DM) technologies, this paper examines the impact of music education on students' psychological health. The study demonstrates that the DM algorithm utilised in this work has the lowest error rate, with an average error rate of only 6.90%, followed by the ACA method with an average error rate of 17.48%, and finally the AI algorithm with an average error rate of 29.35%. As can be shown, this approach is more suited to research the effects of music instruction on students' psychological well-being. The functional module based on DM is developed through simulation experiments to confirm the application effectiveness of the DM algorithm. This is done by using the data source of DM and the structural model of the mining system to build this module on the foundation of the original psychological evaluation system.

## 1. Introduction

The current society is a society with extremely fierce competition for talents. Music can enable people to keep a healthy and clear mind, behave themselves, and actively participate in the process of social development. The essence of music education is to return to humanism and carry out effective teaching strategies according to people's educational needs, which ultimately serves people's growth. Over time, it is easy to evolve into depression. As a generation growing up in a favorable environment, they have become a large special group with poor psychological conditions. Their psychological health problems are mainly manifested as negative life, self-control, low psychological endurance, weak will, difficult to cope with setbacks, and behaviors such as fighting, swearing, lying, weariness of learning, playing truant, mixed life, and serious self-injury or injury [1]. In addition to being a method of art instruction, music education is important in psychological recovery and therapy. Due consideration must be given to the importance and role of music education in the treatment of sickness. We should adapt engaging music-making activities for teaching with the purpose of psychological adjustment based on the reality of students' mental health and widely implement them in the practise of students' psychological health. Middle school children can often learn about different cultures and subdue their emotions by listening to engaging music. Even the process of putting music education into practise is enjoyable. Under its influence, students' pressure from all directions will be lifted, lowering their learning anxiety. Due to the late start and growth of music education in higher vocational colleges, the course settings and instructional strategies are not appropriate. Only a few higher vocational colleges offer organised music education courses, despite the fact that this neglects music education's proper place in raising overall student quality [2]. In the process of getting along with others, we can reflect our own psychological quality, to see whether our communication ability with others is barrier and whether we can freely express our real thoughts. Middle school students who are good at listening to music often have good personalities and can use music to express their own feelings. Music can infect many people and bring some vitality to the boring environment. The nonverbal aesthetic experience of music and the activities of performing music are used to achieve the purpose of psychological adjustment, which has high theoretical value for both music psychology and psychiatry. Simultaneously, various teaching strategies are chosen based on the circumstances of the pupils, enhancing the practical application of music education and broadening its fresh perspective. This study can help advance the field of music psychology and music education theory, which will benefit the growth of music education in China and the discipline's development as a whole.

Therefore, this paper studies the influence of music education on students' psychological health based on DM technology. DM comes from frequent itemsets, and its necessary condition is that the rules in frequent itemsets meet the minimum confidence given by users. The computational complexity of finding association rules is simpler and more intuitive than that of finding frequent itemsets. Therefore, the research on how to improve the efficiency of mining association rules often focuses on the generation of frequent itemsets. The fields generally involved include statistics, pattern recognition, artificial intelligence [3], machine learning [4, 5], database technology, data warehouse technology, and data visualization analysis [6]. The method of data differentiation is used to compare the general characteristics of the target class data object with several comparative class data objects, find their differences, and generate a distinctive description. Concept description is actually to abstract data and find its connotation.

The implementation of music education is not only the infiltration and influence of aesthetic education and moral education, but its inherent positive power is very important for students' physical and mental development. The psychological adjustment of music is not only reflected in the teaching process but also in the follow-up teaching effect, which plays a positive role in students' physical and mental health. Undoubtedly, good music teaching methods can help middle school students enrich their inner emotions and improve their personality charm. It can also enable middle school students to feel the wonder and beauty of the world. Many real data are large-scale data content, and complicated data analysis will consume a lot of time, thus making data analysis infeasible or unrealistic. Although the data set after data reduction is small, it still needs to keep the integrity of the original data set, and the same or almost the same results will be produced after data analysis, which improves the efficiency of DM. [7, 8].

By analysing the psychological data of students in music education and combining the different application directions of the two kinds of algorithms, the data source and the structure model of the mining system are determined. On the basis of the original psychological evaluation system, the function module based on DM is developed through simulation experiments to verify the application effectiveness of the DM algorithm. This paper puts forward two innovations: (1) a DM model of psychological health evaluation in music education is built in this essay. Data selection, data cleaning, data integration, and data transformation are the primary components of data preprocessing, which is a crucial component of DM. Because the real data being investigated contains so many noise data, redundant data, incomplete data, or sparse data, their presence not only impacts the validity of the DM results but also adds to the effort of DM. (2) The main process of DM is discussed. The process of DM can generally be divided into the following five operations: data preparation, DM, result analysis, and knowledge assimilation. Schools should attach importance to the development of music education, improve teachers' music literacy, and promote students' psychological healthy development through music education. Then, the data stored in the normal category database is evaluated. If the evaluation result is inconsistent with the classified result, that is, if the output is abnormal, the data, and the result report will be modified to “abnormal” and transferred to the abnormal category database.

## 2. Related Work

### 2.1. Research on the Relationship between Music Education and Students' Mental Health

Modern students grew up in the era of information explosion, and the unique keen perception of young people made it easy for them to accept new things. Therefore, music education is more acceptable to middle school students than traditional drug therapy, and its therapeutic effect is more obvious. In the unique aesthetic world of music, unconsciously letting middle school students with psychological problems adjust their emotions, relieve their stress, cultivate their sentiments, and perfect their personality has certain guiding value for the psychological health work in schools. Therefore, many literatures on the role of music in maintaining college students' psychological health have emerged in the academic circles, and these literatures constitute the main part of the related literatures in this research.

Pastrana et al. put forward that the rational use of music education can promote the healthy development of students' psychology and cultivate students' sentiment, and its educational effect is profound and lasting. Therefore, teachers should be good at grasping the characteristics of students, infiltrating music education into psychological health education, and constantly looking for effective ways to promote students' psychological health development, so that students' union can grow into talents needed by the society with all-round and healthy development [9]. Job thinks that music is an art that expresses people's inner feelings in an abstract, delicate, and rich way. It is not the expression of concrete things, but the direct simulation and sublimation of human emotions [10]. Su and Lai pointed out that the fundamental task of quality education is to cultivate socialist builders with innovative thinking, while music education can stimulate students' imagination and association, develop students' interests, emotions, and other nonintellectual factors, so as to cultivate students' innovative personality [11]. Silverman and Jennifer put forward that the educational function and effect of music education on cultivating students' sentiment, perfecting their personality, and improving their ideological and moral quality are often beyond the reach of classroom didactic teaching and other educational modes. Some scholars have done in-depth research on the functions of music, and some scholars have pointed out that music has psychological effects such as expression and expression, induction and infection, catharsis and release, and transfer and transformation [12]. Qin et al. show that the psychological health of college students is one of the focuses of the current society, and it is a way worth exploring to use music to adjust the mental state of college students [13]. Kuebel analyzes the psychological problems, communication problems, and love problems encountered by college students during their life and study and helps students to conduct psychological counseling according to scientific emotional management and adjustment, so as to help them build a healthy psychological state. According to the students' personality and psychological characteristics, this paper puts forward five strategies of emotion regulation, and it is a key regulation method to appease the emotion, cheer up the spirit, and release the pressure with the help of music [14]. Lin stated that one can gain a sense of self-control over life through music communication and music activities, alleviate interpersonal conflicts, and establish a good relationship within the family and among peers. Music can change the release of hypothalamic transmitters, regulate the physiological state of endocrine system and autonomic nervous system, and keep human functions in a good physiological state [15]. Yao shows that a good song can make people happy physically and mentally, and playing it at the right time can make a good song play its greatest role. For example, a soothing song in the morning can make students calm down and better cope with the day's learning tasks; a happy song at noon can relax students' nervous psychology; in the evening, a relaxing song can eliminate students' fatigue and relax their brains [16]. Wu indicates that some students are addicted to the Internet, close themselves and escape from reality, which will affect their physical and psychological health over time. And music can draw people closer with its invisible emotional expression [17]. Payne et al. think that the potential psychological adjustment of music is very critical, which not only edifies students' sentiment but also promotes emotional communication among students, makes interpersonal relationships among students more harmonious, cultivates mutual assistance and assistance ability, and promotes students' physical and psychological health development [18].

### 2.2. Research on the Influence of Music Education on Students' Mental Health

The contemporary academic community has done a more thorough study on the mechanism of music education on students' psychological issues as a result of the examination of various research publications mentioned above, which first identified the issues with the current music education system. This study makes an effort to use DM technology to analyse the psychological issues that students are experiencing and offers some ideas for improving and changing music instruction from the standpoint of psychological adjustment. Additionally, it efficiently releases the stress that middle school pupils have built up, accomplishes the ultimate purpose of cleansing their psychology, and effectively averts the aforementioned scenario. One type of art education is music education. It prioritises aesthetics and seeks to develop people's capacity to recognise, express, and produce beauty. Music education serves a crucial role today that other academic fields do not, especially in the context of our ardent advocacy of quality education and aesthetic education. Education in music is crucial for developing willpower. Psychologically, music, as the spiritual food of people, can promote and influence people's spiritual world. Music can awaken people's innermost feelings without any utilitarianism. Music can reactivate those things hidden in people's hearts, change people's subjective knowledge, combine these knowledge, and finally recombine our spiritual world while releasing our emotions. Music has a powerful power to change emotions, which is faster, more powerful, and more direct than any other art form. Music can help us change bad emotions and form new emotional experiences; it also allows us to change our self-awareness and form a new stable personality.

The music education through DM technology not only cultivates the students' music perception ability but also effectively cultivates the students' interest in learning and life. Will is closely related to cognitive emotional activities. It is embodied in the persistence and stability of pursuing ideals and goals and the correct treatment of difficulties and setbacks in learning and life. The scientific and rigorous expression of the relationship between music education in Higher Vocational Colleges and the psychological health of nonmusic majors from the perspective of statistics and case research under the DM technology will more clearly demonstrate the effectiveness of such research.

## 3. Method

### 3.1. Concept and Process of Data Mining

The goal of data mining is to extract knowledge. The original data may be dispersed over the network and may be heterogeneous, semistructured, or structured. Concepts, rules, rules, and patterns are utilised to show the found knowledge and can be used for process control, query optimization, information management, decision assistance, and self-data maintenance. DM originates from frequent itemsets, and one of its prerequisites is that those frequent itemsets' rules satisfy the minimal level of user confidence. Discovering association rules has a lower computational complexity than finding frequent item sets, and it is also more intuitive. As a result, the creation of frequent itemsets is frequently the subject of research on how to make mining association rules more efficient [19]. The amount of data amassed by people in various industries has expanded significantly with the advent of information science and technology. One of the research's main areas of study is how to extract usable knowledge and rules from enormous data. It is a supporting technical method in the DM process. Complex information technologies and mathematical techniques are frequently used in the process of DM. By using graphic, animation, and image methods to carry out operations and direct mining, this technology may be used by users more effectively. It is challenging to adopt DM approaches if these techniques are not used. People believe that DM is the same as knowledge discovery from a pattern processing perspective since it uncovers hidden patterns. The main process of DM is shown in Figure 1.

The process of DM can generally be divided into the following five operations:

*(1) Determine Mining Objects*. We cannot predict the knowledge information finally mined in advance, but we can predict and determine the target tasks to be achieved and the problems to be solved in the initial mining analysis. Through preanalysis of prior knowledge, we can learn relevant industry knowledge in advance, which is conducive to analysis and find out valuable information.

*(2) Data Preparation*. The time spent in this stage occupies most of the DM process. Without this preparation stage, DM will become a blind retrieval process, and the results may become wrong and meaningless. Therefore, the data preparation stage is extremely important for DM.

*(3) DM*. In the previous stage, valuable data sets can be obtained through data selection, data preprocessing, and data conversion. DM is to select the appropriate algorithm to solve this problem for the data set obtained by processing. Most of the work can be completed automatically by the computer, and finally the important rules and knowledge information hidden in the corresponding data can be obtained.

*(4) Result Analysis*. The result analysis is to use the corresponding analysis methods to interpret the model found by the mining and evaluate the mining results according to the mining operation after the DM is completed. If the mining result has redundant or irrelevant knowledge, it needs to be deleted; if it is inconsistent with the original goal, you need to return to the data preparation stage, reselect the data, and create a new analysis model.

*(5) Knowledge Assimilation*. Knowledge assimilation is to integrate the implied valuable knowledge obtained by DM analysis into the corresponding system organization structure, so that it can be applied and tested in the information system.

Music education is a kind of art education. It takes aesthetics as its core and aims to cultivate people's ability to appreciate, express, and create beauty. Today, when we vigorously advocate quality education and aesthetic education, music education has an important function that other disciplines do not have. Music education is equally important to the cultivation of will. DM includes several parts, such as determining the task type of mining, selecting the mining algorithm, and comparing the data. Its purpose is to find potential and useful information from a large amount of data through appropriate DM algorithms and use it in actual production activities, so as to generate more benefits [20]. Although the data set after data reduction is small, it still needs to keep the integrity of the original data set, and the same or almost the same results will be produced after data analysis, which improves the efficiency of DM. By analysing the psychological data of students in music education and combining the different application directions of the two kinds of algorithms, the data source and the structure model of the mining system, are determined.

### 3.2. Application of Data Mining Technology in Psychological Problems of Music Pedagogy Students

In music teaching, teachers are very important. The essence of music education is to return to humanism and carry out effective teaching strategies according to people's educational needs, which ultimately serves people's growth. Over time, it is easy to evolve into depression. As a generation growing up in a favorable environment, they have become a large special group with poor psychological conditions. It can add a touch of aura to middle school students after boring study, thus purifying their psychology. It is very simple for middle school students to listen to music and do some hand in hand, turn around, touch their feet, stomp their feet, etc., and I believe they will feel happiness and joy from it. Let them feel the charm of music in these movements and know the meaning of harmony with others. In addition, we should also understand the collective sense of honor of the group and the awareness of cooperation with others, know how to respect opponents, and assist partners to accomplish their goals and tasks better and faster. Schools should attach importance to the development of music education, improve teachers' music literacy, and promote students' psychological healthy development through music education. After then, analyse the information from the usual category database. The data and result report will be changed to “abnormal” and added to the database for the abnormal category if the evaluation results are contradictory with the classified findings, or if the output is abnormal [21]. Data preprocessing, which includes data selection, cleansing, integration, normalisation, and transformation, is a crucial component of DM. Since the real data to be investigated contains a lot of noisy data, redundant data, incomplete data, or sparse data, their presence not only impairs the conclusions' veracity but also adds to the workload of DM [22, 23]. Therefore, through DM technology, this paper extracts useful information from a large number of students' psychological health evaluation databases, which can be used as a reference for the prediction of higher vocational students' mental problems. The detailed model structure diagram is shown in Figure 2.

#### 3.2.1. Data Acquisition

After the objectives and objects of mining are clear, the next step is to study and analyse the data sources used. Psychologically, music, as the spiritual food of people, can promote and influence people's spiritual world. Music can awaken people's innermost feelings without any utilitarianism. Music can reactivate those things hidden in people's hearts, change people's subjective knowledge, combine these knowledge, and finally recombine our spiritual world while releasing our emotions. Specifically, 260 freshmen and sophomores were selected, including 157 males and 103 females. The psychological assessment database of the involved vocational colleges is stored and managed by SQL Server 2008. The personal information mainly includes gender, age, major, place of origin, family economic income, and individual social support utilization, with a total of 6 items. SCL-90 includes 90 assessment items and 10 factor scores. Each item adopts a five-level scoring system. The higher the score, the more serious the symptom.

#### 3.2.2. Data Preprocessing

The data information obtained by preprocessing the data source may be inaccurate, partial, imprecise, repetitious, and useless when the previous procedure is complete. It cannot currently be utilised directly for mining analysis. So that they have the same meaning and expression, it is now important to standardise the data from various structures in various data sources. An essential step in the DM process is data preparation. Many erroneous noise data will be produced when processing linked data owing to a variety of circumstances. Noise data preprocessing can significantly increase mining productivity, and speed up subsequent analysis. As a result, the information used in this article has 11 dimensions.

*T* is the sum of the scores of 90 projects, and *T*_*i*_ is equal to the total score of each project that constitutes this factor divided by the number of projects, namely

(1) $$\begin{array}{c} T=\overset{90}{\underset{x=1}{\sum }}t=\overset{10}{\underset{i=1}{\sum }}t_{im},\\ T_{\alpha }=\frac{T}{90},\\ T=\frac{1}{n}\overset{n}{\underset{m=1}{\sum }}t_{im}. \end{array}$$

Let node *N* store all samples of data partition *D*. The expected information needed to classify samples in *D* is given by the following formula:

(2) $$\begin{array}{c} Info\left(D\right)=-\overset{m}{\underset{i=1}{\sum }}\log\left(p_{i}\right), \end{array}$$

where *p*_*i*_ is the probability that any sample in *D* belongs to *C*_*i*_, which is calculated by (*C*_*i*,*D*_)/(*D*).

The expected information required for classifying samples of *D* based on attribute *A* can be obtained by the following formula:

(3) $$\begin{array}{c} {\text{Info}}_{A}\left(D\right)=\overset{v}{\underset{j=1}{\sum }}\times \text{Info}\left(D\right), \end{array}$$

where *Info*_*A*_(*D*) is the expected information needed to classify the samples of *D* according to the attribute *A*.

Knowing the value of attribute *A* leads to the decrease of entropy, which can be obtained by the following formula:

(4) $$\begin{array}{c} \text{Gain}\left(A\right)=\text{Info}\left(D\right)-\inf o_{A}. \end{array}$$

In actuality, classification is the process of removing information from a system to lessen system confusion and let the system develop in a more predictable, ordered, and systematic manner.

The information gain rate is defined as follows:

(5) $$\begin{array}{c} \text{Gain}=\frac{\text{Gain}\left(A\right)}{\text{SplitInfo}}. \end{array}$$

To normalise the information obtained, split information is used in the formula. Similar to *Info*(*D*), split information is defined as

(6) $$\begin{array}{c} \text{SplitInfo}\left(D\right)=-\overset{v}{\underset{j=1}{\sum }}\log2\frac{D_{j}}{D}, \end{array}$$

where SplitInfo(*D*) represents information generated by dividing the training sample set *D* into *v* plans corresponding to *v* outputs of the attribute *A* test.

Even though not all of the samples in this branch fall under the same category, the error substitution rate formula can be used if the number of samples in each category is very different.

(7) $$\begin{array}{c} \text{pure}=\frac{n-n^{\prime }}{m}, \end{array}$$

where *n* represents the number of samples on a branch, *n*′ represents the number of samples in most categories on the branch, and *m* represents the total number of samples in the training sample set.

If established, *T*_*t*_ will be cut off and replaced with corresponding leaves and will be defined as

(8) $$\begin{array}{c} SE=\sqrt{\frac{e\left(T_{t}\right)\left[n\left(t\right)-e^{\prime }\left(T_{t}\right)\right]}{n\left(t\right)}}. \end{array}$$

Therefore, this algorithm is faster and better than other algorithms and is recognized as one of the most accurate pruning algorithms. Good music education can guide college students to form correct values, world outlook, and outlook on life. To enjoy music is not only to listen to music but also to feel the artistic conception and experience the spirit and significance of the music works. Music education can enable students to better understand the different beauty under the background of each era, so that they can achieve comprehensive and healthy development. The achievements of music education in playing its psychological adjustment function help more students regain confidence and happiness and actively integrate into the collective life and feel the happiness brought by music education. Music educators also actively play the function and value of music education in teaching activities, promote the comprehensive development of students' quality and ability, and help them find a sense of happiness and belonging.

## 4. Results Analysis and Discussion

As shown in Table 1 and Figure 3, among the four propositions of status recognition, music education should not be placed in a relatively secondary position of education of other disciplines (a), music education should be placed in an equal position of education of other disciplines (b), other education of perception should not be placed above music education (c), and music education should not be replaced by music education (d). The proposition of “music education is indispensable and irreplaceable” has the highest recognition, and 95 (75.2%) of the teachers interviewed chose the option of “very agree” to “Music education should be in the same position as other education”, and the frequency and proportion of respondents who choose “very agree” are second, with a value of 86 (72.5%); the relatively low recognition is that “education of other disciplines should not be superior to music education”, and the frequency and proportion of “very agree” is 74 (60.5%).

The title is “music education should not be placed in a relatively secondary position in education of other disciplines”. A total of 114 valid data were obtained and 8 items were missing. Among them, the frequency of choosing “very agree” and “disagree” was 85 (69.5%) and 2 (10.3%), respectively, and the frequency of choosing “very disagree” was 2 (20.2%) as shown in Table 2.

The title is “Why you don't like music lessons”, and the answer to the option “Afraid of affecting the study of cultural courses” reflects students' attitude towards the status of music education. The test questions are multiple choices, and a total of 982 valid data are obtained. The frequency of choosing this option has reached, as shown in Table 3.

The radar chart is prepared according to the table data, as shown in Figure 4. According to the following three categories, the teacher's lectures are not attractive (I), useless (II), and afraid of affecting the study of cultural courses (III), as shown in Figure 4. Obviously, the option of “fear of affecting the study of cultural courses” accounts for the largest proportion of “reasons for not liking music courses”, reflecting the attitude of the interviewed students that music courses are secondary to cultural courses.

As shown in Figure 5, the age distribution of full-time music teachers is most concentrated in the age group of 26-35 years old, with the highest proportion of 17.1%; the second is under 26 years old and 23-26 years old, accounting for 9.5% and 13.2%, respectively. Taking the age of 38 as a dividing line, 72.5% of the full-time music teachers are under the age of 38. Over the age of 38, the proportion of teachers in all age groups has dropped sharply, including 7.1% of full-time music teachers aged 38-41, 7.8% of full-time music teachers aged 44-50, and 6.7% of full-time music teachers over 50. It can be said that the full-time music teachers in the interviewed rural schools are generally younger.

In accordance with the analysis of teachers' teaching ages based on analyses of age structures, as shown in Figure 6, the fraction of music teachers with teaching ages under 16 is around 74.5%, further limiting the scope to music teachers with teaching ages under 14 years. A total of 58.7% of the instructors that were questioned belong to this group of educators. In summary, it can be inferred from the analysis above that the age distribution of the music teachers in the rural schools where they were interviewed is young, that there is a flaw in the distribution of full-time and part-time music teachers, but that the two can still work in harmony, and that the average age of music teachers is relatively young.

The three methodologies used in this experiment to examine the impact of music education on students' psychological health are artificial intelligence (AI), ant colony algorithm (ACA), and differential evolution (DM) algorithms. In Figure 7, the experimental outcomes are displayed.

According to the data in Figure 7, the DM algorithm used in this study has the lowest error rate of the three, with an average error rate of just 6.90%. The ACA algorithm comes in second with an average error rate of 17.48%, and the AI algorithm comes in third with an average error rate of up to 29.35%. This approach is therefore better suited to research on how music education affects students' psychological well-being.

## 5. Conclusion

As long as it is managed properly, music education, whether it be formal music instruction or artistic practise related to music, is a significant way to cultivate college students' psychological wellness. College students can engage in aesthetic and scene experiences through music performance and music appreciation activities, and they can work with mental health education, mental health counseling, and mental health psychotherapy to jointly increase college students' level of mental health. The impact of music education on students' psychological health is examined in this article using DM technology. According to the research, the DM algorithm used in this paper has the lowest error rate, with an average error rate of just 6.90%. The ACA algorithm comes in second with an average error rate of 17.48%, and the AI algorithm comes in third with an average error rate of 29.35%. The research of the impact of music education on students' psychological health is therefore more suited for this methodology. Kids can purify their hearts, grow their emotions, and attach value to music education with the use of DM technology-based music education, which can also help students liberate their beautiful hearts. This not only improves the methods of music instruction but it also plays a significant role in reducing student stress and fostering the development of sound psychological and personal traits in college students. Cognitive emotional processes are directly tied to will. The steadfastness with which one pursues principles and objectives, as well as the appropriate response to challenges and failures encountered in both learning and life, are examples of this.

## Figures and Tables

**Figure 1:** Main process of DM.

**Figure 2:** DM model of psychological health assessment in music education of students.

**Figure 3:** Understanding of the status of music education.

**Figure 4:** Reasons why students dislike music lessons.

**Figure 5:** Age distribution of full-time and part-time music teachers.

**Figure 6:** Cross distribution of teaching age and music course teaching age.

**Figure 7:** Error rate of the influence of music education on students' psychological health.

**Table 1:** General table of recognition frequency of school music education status.

		Response		Percentage of cases
		*N*	Percentage	
Understanding of the position of music education in school education	Very agree.	340	75.2%	300.0%
	Disagree	90	14.4%	6.3%
	Very disagree	50	10.4%	0.8%

Total		480	100.0%	307.1%

**Table 2:** Should not be in a secondary position to know the frequency table.

		Frequency	Percentage	Effective percentage	Cumulative percentage
	Very agree	85	69.5	73.8	100.0
	Disagree	2	10.3	0.9	1.9
	Very disagree	2	20.2	0.9	0.9

Defect	System	8	5.9		

Total	122		100.0		

**Table 3:** Reasons why I do not like music lessons frequency table.

		Response		Percentage of cases
		*N*	Percentage	
Why I do not like music lessons	The teacher's lecture is not attractive	342	25.6%	24.7%
	It is no use learning	175	20.2%	12.8%
	Afraid of affecting cultural studies	465	54.2%	33.7%

Total		982	100.0%	

## Data Availability

The data used to support the findings of this study are available from the corresponding author upon request.

## References

[1] Zhang T., Liu S. (2021). Evaluation of the effect of music education on improving students' psychological health based on intelligent fuzzy system. *Journal of Intelligent and Fuzzy Systems*.

[2] Zhiqiao L. I., Center A. (2018). A study of new-style music promoting the psychological health of college students. *Journal of Educational Science of Hunan Normal University*.

[3] Zhao M., Liu Q., Jha A. VoxelEmbed: 3D instance segmentation and tracking with voxel embedding based deep learning.

[4] Ding Y., Zhang Z., Zhao X. (2022). Self-supervised locality preserving low-pass graph convolutional embedding for large-scale hyperspectral image clustering. *IEEE Transactions on Geoscience and Remote Sensing*.

[5] Gu X., Cai W., Gao M., Jiang Y., Ning X., Qian P. (2022). Multi-source domain transfer discriminative dictionary learning modeling for electroencephalogram-based emotion recognition. *IEEE Transactions on Computational Social Systems*.

[6] Zhang J., Feng W., Yuan T., Wang J., Sangaiah A. K. (2022). SCSTCF: spatial-channel selection and temporal regularized correlation filters for visual tracking. *Applied Soft Computing*.

[7] Samanta A., Joglekar A. (2017). Crime classification and criminal psychology analysis using DM. *Journal of Intelligent and Fuzzy Systems*.

[8] Zhang X., Luo P. (2021). Analysis of psychological education factors based on computer software and hardware collaboration and DM. *Music Educators Journal*.

[9] Pastrana J. L., Reigal R. E., Morales-Sánchez V. (2019). Data mining in the mixed methods: application to the study of the psychological profiles of athletes. *Frontiers in Psychology*.

[10] Job M. A. (2018). DM techniques applying on educational dataset to evaluate learner performance using cluster analysis. *Transportation Research Part F: Traffic Psychology and Behaviour*.

[11] Su Y. S., Lai C. F. (2021). Applying educational data mining to explore viewing behaviors and performance with flipped classrooms on the social media platform Facebook. *Frontiers in Psychology*.

[12] Silverman M. J., Jennifer B. (2018). Acute care mental health workers' assumptions and expectations of music therapy: a qualitative investigation. *Arts in Psychotherapy*.

[13] Qin H., Wu Z., Wang M. (2020). Application of data mining in cultivation of student mental health. *IOP Conference Series Materials Science and Engineering*.

[14] Kuebel C. (2019). Health and wellness for in-service and future music teachers: developing a self-care plan. *Music Educators Journal*.

[15] Lin Y. I. (2017). On the function and method of music education in psychological health of undergraduates in science and technology universities. *Journal of North China Institute of Science and Technology*.

[16] Yao C. G. (2017). Effect analysis on music therapy to secondary vocational student's psychological health. *Education Teaching Forum*.

[17] Wu X. (2017). Psychological therapy in "seven elicitation" and psychological health education of middle school students. *The Science Education Article Collects*.

[18] Payne P. D., Lewis W., Mccaskill F. (2020). Looking within: an investigation of music education majors and mental health. *Journal of Music Teacher Education*.

[19] Rawlings J. R., Espelage D. L. (2020). Middle school music ensemble participation, homophobic name-calling, and mental health. *Youth & Society*.

[20] Rodgers D. (2018). London review of education community music as a vehicle for tackling psychological health- related stigma. *rScroll*.

[21] Gora M., Sexton-Radek K. (2018). Music and psychological health. *rScroll*.

[22] Rebecchini L. (2021). Music, mental health, and immunity. *Brain, Behavior, & Immunity - Health*.

[23] Yin Z. (2021). Research on the application of music-based psychological adjustment in improving postgraduates' psychological health. *Revista Brasileira de Medicina do Esporte*.

